# γ-tocotrienol prevents 5-FU-induced reactive oxygen species production in human oral keratinocytes through the stabilization of 5-FU-induced activation of Nrf2

**DOI:** 10.3892/ijo.2015.2849

**Published:** 2015-01-26

**Authors:** HIDEYUKI TAKANO, YUKIHIRO MOMOTA, KOUICHI KANI, KEIKO AOTA, YOSHIKO YAMAMURA, TOMOKO YAMANOI, MASAYUKI AZUMA

**Affiliations:** Department of Oral Medicine, Institute of Health Biosciences, The University of Tokushima Graduate Faculty of Dentistry, Tokushima, Japan

**Keywords:** oral keratinocytes, oral cancer, mucositis, reactive oxygen species, 5-FU, γ-tocotrienol, Nrf2

## Abstract

Chemotherapy-induced oral mucositis is a common adverse event in patients with oral squamous cell carcinoma, and is initiated through a variety of mechanisms, including the generation of reactive oxygen species (ROS). In this study, we examined the preventive effect of γ-tocotrienol on the 5-FU-induced ROS production in human oral keratinocytes (RT7). We treated RT7 cells with 5-FU and γ-tocotrienol at concentrations of 10 μg/ml and 10 nM, respectively. When cells were treated with 5-FU alone, significant growth inhibition was observed as compared to untreated cells. This inhibition was, in part, due to the ROS generated by 5-FU treatment, because N-acetyl cysteine (NAC), a ROS scavenger, significantly ameliorated the growth of RT7 cells. γ-tocotrienol showed no cytotoxic effect on the growth of RT7 cells. Simultaneous treatment of cells with these agents resulted in the significant recovery of cell growth, owing to the suppression of ROS generation by γ-tocotrienol. Whereas 5-FU stimulated the expression of NF-E2-related factor 2 (Nrf2) protein in the nucleus up to 12 h after treatment of RT7 cells, γ-tocotrienol had no obvious effect on the expression of nuclear Nrf2 protein. Of note, the combined treatment with both agents stabilized the 5-FU-induced nuclear Nrf2 protein expression until 24 h after treatment. In addition, expression of Nrf2-dependent antioxidant genes, such as heme oxygenase-1 (*HO-1*) and NAD(P)H:quinone oxidoreductase-1 (*NQO-1*), was significantly augmented by treatment of cells with both agents. These findings suggest that γ-tocotrienol could prevent 5-FU-induced ROS generation by stabilizing Nrf2 activation, thereby leading to ROS detoxification and cell survival in human oral keratinocytes.

## Introduction

Oral mucositis is a common adverse event in chemotherapy and radiotherapy against human head and neck cancers (1,2), and results from the damage of the mucosal lining of the gastrointestinal tract, especially the oral and oropharyngeal mucosa (3). Previously, mucositis was considered to arise as a consequence of epithelial injury (4–6), i.e., it was thought that chemotherapy and radiotherapy non-specifically kill the rapidly proliferating cells of the basal cell layer, thereby abolishing the ability of the layer to renew itself. In the case of radiotherapy-induced mucositis, the cell death was attributed to DNA strand breaks in the oral basal epithelial cells, while in chemotherapy-induced mucositis it was attributed to direct basal cell damage (non-DNA injury) caused by the drugs permeating the cells from the submucosal blood supply (3).

Although the clinical symptoms of oral mucositis, such as ulceration of the mucosal epithelium, pain, infection, and swallowing dysfunction, are almost all the results of epithelial injury (7), accumulating evidence indicate that the clinical manifestations of this condition are attributable to a series of interactive biological events that involve all of the cells and tissues of the mucous membrane (8–10). For example, morphological observations suggest that damage in the submucosal endothelium and connective tissue occur first, followed by injury of the epithelial cells (9). Moreover, it has been reported that endothelial damage (endothelial toxicity) might be the initiating event in the radiotherapy-induced mucositis (10), indicating that several chemotherapeutic agents, including 5-FU and cisplatin, also similarly exert their endothelial toxicity (11,12). Therefore, chemotherapy- and radiotherapy-induced oral mucositis is initiated by direct damage to basal epithelial cells and cells in the underlying tissues.

Chemotherapy induces non-DNA damage in the cells, e.g., basal epithelial cells, through a variety of mechanisms, some of which are mediated by the generation of reactive oxygen species (ROS) (13). Although a moderate increase in ROS can promote cell proliferation and differentiation (14,15), excessive amounts of ROS can cause oxidative damage to lipids, proteins and DNA (16), thereby leading to cell death or abnormal cell growth (17). Maintenance of the ROS level in cells is thus crucial for normal growth and survival. To achieve such maintenance, the cells control ROS levels by balancing ROS generation with their elimination by ROS-scavenging systems such as intracellular redox-balancing genes [heme oxygenase-1 (*HO-1*)], phase II detoxifying genes [NAD(P) H:quinone oxidoreductase-1 (*NQO-1*)], and genes encoding transporters (multidrug resistant proteins) (18). Many of these genes contain an enhancer sequence known as the antioxidant response element (ARE) (19–21), and are enhanced by the transcription factor NF-E2-related factor 2 (Nrf2). Based on the functions of these ARE-containing genes, it seems likely that activation of Nrf2 target genes would stimulate the detoxication of xenobiotics, such as chemopreventive drugs, and protect cells from ROS-driven apoptosis (22).

A vitamin E constituent may be one such candidate agent derived from natural sources with great potential for preventing the cell death induced by anticancer drugs. Vitamin E is a general term representing a family of compounds that is further divided into two subgroups: tocopherols and tocotrienols (23). Although tocopherols and tocotrienols exist in α, β, γ and δ form, the two differ structurally in that tocopherols contain a saturated phytyl chain, whereas tocotrienols possess an unsaturated side chain. Thus far, tocopherols have been studied extensively, while very little is known about tocotrienols. Previous studies including ours have shown that tocotrienols are more potent antioxidant agents than tocophenols (24), and that γ-tocotrienol enhances the chemosensitivity of human oral cancer cells to docetaxel (25). Importantly, γ-tocotrienol exerts significant anti-proliferative effects in malignant cells, but not in normal cells (26). Therefore, it is likely that the oral mucositis caused by chemotherapeutic agents could be prevented by a low dose of γ-tocotrienol through the detoxification of ROS in basal epithelial cells.

In the present study, we demonstrate that simultaneous treatment of human oral epithelial (RT7) cells with 5-FU and γ-tocotrienol suppressed the 5-FU-induced generation of ROS, leading to the amelioration of cell growth. We also found that the inhibition of ROS generation in RT7 cells was due to the stabilization of 5-FU-mediated activation of Nrf2, which resulted in the enhanced production of the ROS-scavenging enzymes HO-1 and NQO-1.

## Materials and methods

### Cells and media

RT7, an immortalized human oral keratinocyte cell line, was established by transfection of human telomerase reverse transcriptase (hTERT) and E7, as previously described (27), and the metastatic human oral cancer cell line (B88) was previously established in our laboratory (28). RT7 and B88 cells, respectively, were cultured in keratinocyte serum-free medium (SFM) (Gibco-BRL, Gaithersburg, MD, USA) that included 25 μg/ml bovine pituitary extract, 0.05 ng/ml epidermal growth factor, 100 U/ml penicillin and 100 μg/ml streptomycin, and in DMEM supplemented with 10% fetal bovine serum (both from Gibco-BRL), 100 U/ml penicillin and 100 μg/ml streptomycin in the presence of 5% CO_2_ in an incubator at 37°C.

### In vitro cell growth assay

Cells (3×10^3^ cells/well) were grown on 96-well plates (Falcon; Becton-Dickinson Labware, Lincoln Park, NJ, USA) in SFM and DMEM in the presence or absence of 5-FU (1, 2, 5, 10 μg/ml) (Taiho Pharmaceutical Co., Ltd., Tokyo, Japan) and γ-tocotrienol (10 nM) (with a purity exceeding 98.7%; Eisai Food & Chemical Co., Tokyo, Japan) alone, or both for 3 days. In addition, RT7 cells were also treated with 5-FU and a ROS scavenger, N-acetyl cysteine (NAC) (Sigma-Aldrich, St. Louis, MO, USA), to inhibit ROS generation. Thereafter, 10 μl of 5 mg/ml 3-(4,5-dimethyl-thiazol-2-yl)-2,5-diphenyltetrazolium bromide (MTT) were added to each well and the cells were incubated for 4 h. The blue dye taken up by the cells was dissolved in dimethyl sulfoxide (100 μg/ml), and the absorbance was measured with a Titertek Multiscan spectrophotometer (Flow Laboratories, Irvine, UK) at 570 nm. All assays were run in triplicate.

### Measurement of ROS

2′,7′-Dichlorofluorescein diacetate (H_2_DCF-DA; Molecular Probes, Eugene, OR, USA) was used to analyze the intracellular ROS level. RT7 cells were incubated with 5-FU, NAC, or γ-tocotrienol alone, or with a combination of 5-FU and NAC for 48 h. Adherent cells were washed with PBS and stained with 2 μM DCFH-DA diluted in PBS at 37°C in the dark for 30 min (29). The DCFH-DA dye oxidized by ROS can be excited by a 488-nm laser. RT7 cells were washed twice with PBS before flow cytometric analysis using a FACSCalibur flow cytometer and data were analyzed by CellQuest software (both from Becton-Dickinson, East Rutherford, NJ, USA).

### Nuclear and cytosolic extract preparations

RT7 cells were seeded on 100-mm plastic petri dishes (Falcon; Becton-Dickinson Labware). Twenty-four hours after seeding, the cells were treated with either 5-FU, γ-tocotrienol, or both for 24 h, and then the nuclear extracts were obtained according to a previously described method (30). The cells were washed twice with ice-cold PBS before being resuspended in 400 μl of ice-cold lysis buffer consisting of 10 mM N-2-hydroxyethylpiperazine-N′-2-ethanesulfonic acid (HEPES) (pH 7.9), 10 mM KCl, 0.1 mM ethylenediaminetetraacetate (EDTA), 0.1 mM ethylene glycol-bis (2-aminoethylether)-N,N,N′,N′-tetraacetic acid (EGTA), 0.5 mM dithiothreitol (DTT), 0.5 mg/ml benzamidine and 2 mg/ml aprotinin for 15 min. Nonidet P-40 was added to a final concentration of 0.3%, and the lysates were vortexed before being pelleted in a microfuge. The supernatants of this centrifugation were designated cytosolic extracts. Each nuclear pellet was resuspended in 50 μl of extraction buffer consisting of 10 mM HEPES (pH 7.9), 400 mM NaCl, 10 mM KCl, 0.1 mM EDTA, 0.1 mM EGTA, 1 mM DTT, 0.5 mM phenyl-methylsulfonyl fluoride and 2 mg/ml aprotinin and then placed on ice for 30 min. The nuclear extracts were pelleted, and the supernatants were designated nuclear extracts. The protein concentrations contained in samples were determined using a Bio-Rad protein assay kit (Bio-Rad, Hercules, CA, USA).

### Western blot analysis of Nrf2, Kelch-like ECH-associated protein 1 (Keap1) and β-actin proteins

Cytosolic extracts (20 μg) were subjected to electrophoresis on 10% SDS-polyacrylamide gels, then transferred onto nylon membranes. The membranes were blocked with 3% bovine serum albumin and incubated with each of the following antibodies (all from Santa Cruz Biotechnology, Inc., Santa Cruz, CA, USA): anti-Nrf2, anti-Keap1 and anti-β-actin. After intervening rinses with PBS, the antibodies were detected using a chemiluminescence western blot analysis kit (Amersham Pharmacia Biotech, Tokyo, Japan) according to the manufacturer’s instructions.

### Immunofluorescence staining for Nrf2 protein

Cells grown on coverglasses were washed with PBS three times, fixed in acetone at 4°C for 10 min, and incubated for 1 h at 37°C with mouse polyclonal antibody to Nrf2 (Abcam, Cambridge, MA, USA) at a dilution of 1:200. After three rinses with PBS, the coverglasses were incubated for 1 h with fluorescein-conjugated goat anti-mouse IgG (1:200 dilution; Abcam). The coverglasses were then mounted with PermaFluor™ Aqueous Mounting Medium (Lab Vision Corporation, Fremont, CA, USA). To establish a negative control, the primary antibody was omitted.

### RNA isolation and quantitative real-time PCR

Total cellular RNA was isolated after the RT7 cells were treated with TRIzol reagent plus 5-FU, or γ-tocotrienol or both (Invitrogen Life Technologies, Carlsbad, CA, USA). The cDNA was synthesized from 5 μg of total RNA using an Advantage cDNA PCR kit (Clontech Laboratories, Inc., Palo Alto, CA, USA). For the quantitative real-time PCR, equal aliquots (1 μl) of cDNA were amplified according to the manufacturer’s TaqMan universal (50 μl) PCR master mix protocol using an ABI PRISM 7300 RT-PCR system (Applied Biosystems Japan, Ltd., Tokyo, Japan). The primer set and TaqMan probe mixture used for the PCR were purchased from Applied Biosystems Japan, Ltd. (HO-1: Hs01110250_m1; NQO-1: Hs02512143_s1). The data were normalized using RT-PCR β-actin primers (Hs99999903_m1; Applied Biosystems Japan, Ltd.)

### Statistical analysis

The statistical analysis was performed using the Mann-Whitney U test; P<0.05 was considered to indicate statistical significance.

## Results

### Optimal concentration of 5-FU used in this study

The concentrations of chemotherapeutic drugs, including 5-FU, used in the clinical setting would be determined based on the balance between the cytotoxicity to cancer cells and non-cytotoxicity to normal cells. Therefore, in this study, we used an immortalized normal human oral keratinocyte (RT7) and a human oral cancer cell (B88) line to determine the optimal dose of 5-FU in our system. The growth inhibitory response of both cell lines to 5-FU was investigated by MTT assay for 3 days. As shown in Fig. 1, 5-FU at the concentrations of 5 and 10 μg/ml had a significant cytotoxic effect on B88 cells, inducing an apparent growth inhibitory response as compared to that in untreated cells, whereas the same concentrations of 5-FU did not exert cytotoxic or cytostatic effects on RT7 cells. Based on this finding, we chose a 5-FU concentration of 10 μg/ml for the use in this study.

### Growth-suppressive effect of 5-FU on RT7 cells via ROS generation

To determine whether or not the 5-FU treatment would stimulate ROS generation in RT7 cells, we measured the levels of ROS using the ROS detection dye DCFH-DA. No increase in ROS was detected at 24 h after treatment with 10 μg/ml of 5-FU (Fig. 2A). Further incubation with 10 μg/ml of 5-FU for 48 h resulted in a significant increase in ROS production in RT7 cells. To examine whether NAC, a ROS scavenger, actually abolishes ROS, we measured the ROS level using the method described above. When RT7 cells were treated with both 5-FU and NAC (0.1 mM) for 24 h, the generation of ROS was not affected. However, ROS production was significantly suppressed at 48 h after treatment with NAC (Fig. 2B). Since ROS affects the suppression of cell growth, we examined the effect of NAC on the growth of RT7 cells. As shown in Fig. 2C, although NAC alone did not affect the growth of RT7 cells, the cell growth that was suppressed by 5-FU was significantly restored through the elimination of ROS in RT7 cells. Therefore, these results indicate that growth suppression by 5-FU may be at least partly due to the generation of ROS from RT7 cells.

### Amelioration of 5-FU-induced growth suppression by γ-tocotrienol via ROS inhibition

The growth response of RT7 cells to γ-tocotrienol (10 nM) was investigated by MTT assay for 3 days. As can be seen in Fig. 3A, γ-tocotrienol alone did not affect RT7 cell growth when compared to the growth of the control cells. Whether or not γ-tocotrienol can restore the suppressive effect of 5-FU on RT7 cell growth was also examined. The dose of γ-tocotrienol (10 nM) that did not affect cell growth when used alone resulted in an enhanced recovery of cell growth when used in combination with 5-FU. In addition, although 5-FU alone stimulated the generation of ROS in RT7 cells, combined treatment with 5-FU and γ-tocotrienol significantly inhibited the production of ROS at 48 h (Fig. 3B).

### Effect of 5-FU and γ-tocotrienol on the expression of Nrf2 and Keap1 proteins

We examined the expression of the proteins Nrf2, a master transcriptional factor of various cytoprotective genes against oxidative stress, and Keap1, a negative regulator of Nrf2, by treatment with 5-FU, γ-tocotrienol, or both. As shown in Fig. 4A, 5-FU induced the nuclear accumulation of Nrf2 in RT7 cells for up to 12 h; however, no apparent effect was observed in γ-tocotrienol-treated cells. Of note, the simultaneous treatment of cells with 5-FU and γ-tocotrienol led to sustained nuclear accumulation of Nrf2 for up to 24 h. As shown in Fig. 4B, the expression of Keap1 was inversely correlated with that of Nrf2: 5-FU inhibited Keap1 expression at 6 and 12 h after treatment, followed by reappearance at 24 h. Although γ-tocotrienol had no effect on the expression of Keap1 in RT7 cells, combined treatment of cells with 5-FU and γ-tocotrienol suppressed the expression of Keap1 for up to 24 h after treatment. Therefore, the sustained activation of 5-FU-induced Nrf2 expression may have been due to the continuous degradation of Keap1 through the combined treatment with 5-FU and γ-tocotrienol in RT7 cells.

### Expression of HO-1 and NQO-1 mRNA by treatment with 5-FU and γ-tocotrienol

To examine the effect of 5-FU and γ-tocotrienol on the expression of the detoxifying enzymes HO-1 and NQO-1 in RT7 cells, we used quantitative RT-PCR analysis. As shown in Fig. 5A and B, although 5-FU treatment at 12 h was associated with a significant increase in the expression of these enzymes, the expression of both enzymes was remarkably suppressed when 5-FU treatment was continued for up to 24 h. When γ-tocotrienol was used, no significant changes were observed in the mRNA expression levels of these enzymes. Importantly, combined treatment of cells with 5-FU and γ-tocotrienol increased the expression levels of HO-1 and NQO-1 mRNA for up to 24 h. These results indicate that expression of the detoxifying enzymes HO-1 and NQO-1 is likely regulated by a master regulatory transcription factor, Nrf2 (31).

## Discussion

Oral mucositis is a common adverse event caused by antineoplastic radiation (radiotherapy) and drug therapies (chemotherapy) for patients with head and neck cancer, and is associated with severe adverse symptomatic health and economic outcomes (32,33). Thus far, although understanding of the pathobiology of this unfavorable condition has increased rapidly over the past decade, there remains no effective way to prevent or treat mucositis (3). Therefore, the objective of the present study was to investigate whether or not γ-tocotrienol, a component of vitamin E, can improve the cell survival of human oral keratinocytes against 5-FU-induced cell toxicity. The results showed that γ-tocotrienol suppressed the 5-FU-induced generation of ROS, leading to the potentiation of RT7 cell growth, and sustained the upregulated expression of Nrf2 by 5-FU, as well as the expression of the detoxifying enzymes HO-1 and NQO-1.

A key challenge to the development of drugs for ameliorating chemotherapy- and radiotherapy-induced oral mucositis is to ensure that they target normal tissue effectively, but do not diminish the tumoricidal effect of the antineoplastic drugs. Therefore, we investigated the optimal concentrations of 5-FU and γ-tocotrienol using human oral cancer cells and normal human oral keratinocytes, and determined that concentrations of 10 μg/ml and 10 nM, respectively, were most effective. Although the concentrations of drugs used in this study showed no significant cytotoxic effects on the growth of normal keratinocytes, the growth of cancer cells was clearly suppressed. At present, several possible mechanism-based treatments for oral mucositis are undergoing trial (3). Some of these approaches target ROS, which are ubiquitous in the tissues of mucosal injury, for cytoprotective intervention in the oral mucosa (34). Thus, we analyzed the effects of a free-radical scavenger, γ-tocotrienol, for its ability to reduce ROS levels. Our results showed that γ-tocotrienol could reduce 5-FU-induced ROS generation, leading to the sustained survival of oral keratinocytes.

Chemotherapy induces non-DNA injury in the epithelial cells through a variety of mechanisms, some of which are mediated by the generation of ROS (3). ROS also activate several injury-producing pathways, such as the nuclear factor-κB (NF-κB) and p53 pathways, in epithelial cells (35). In the present study, we demonstrated that γ-tocotrienol could suppress 5-FU-induced ROS generation, which in turn suggested that γ-tocotrienol induced the inhibition of NF-κB in RT7 cells. Since we have previously shown that γ-tocotrienol suppressed the activation of NF-κB induced by a chemotherapeutic agent (docetaxel) in oral cancer cells (25), mechanism involved in the cell survival of RT7 by γ-tocotrienol might involve regulation of the balance between NF-κB-related pro-apoptotic and anti-apoptotic genes (3).

Cell membrane-bound molecules released during chemotherapy (lipid peroxidation) also result in the upregulation of genes, including those encoding c-Jun and c-Jun amino-terminal kinase (JNK) (35,36). Therefore, these molecules upregulate other transcription factors, such as Nrf2 (37). In addition, it is well known that many chemotherapeutic agents are able to stabilize the expression of Nrf2 by inhibiting Nrf2 degradation, and thereby enhance the protein level of Nrf2 and activate the Nrf2-dependent antioxidant response (38,39). In this study, we have shown that although 5-FU treatment of RT7 cells actually resulted in the activation of Nrf2 for up to 12 h, the combined treatment with 5-FU and γ-tocotrienol led to the sustained activation of Nrf2 for up to 24 h. In addition, the expression of Keap1, an E3 ubiquitin ligase that promotes proteasome-dependent degradation of Nrf2 (40), was inhibited by the 24 h combination treatment, indicating that γ-tocotrienol could activate Nrf2 by suppressing the expression of Keap1 in RT7 cells. Consistent with the above results, a previously reported quantitative RT-PCR analysis clearly demonstrated that expression of the antioxidant enzymes HO-1 and NQO-1 was Nrf2-dependent (41), suggesting that the improved survival of RT7 cells was attributable to the sustained reduction of ROS by γ-tocotrienol.

In conclusion, the results of the present study indicate that γ-tocotrienol potentiates and sustains the 5-FU-induced expression of Nrf2 in human keratinocytes, leading to the continuous degradation of 5-FU-generated ROS via the augmented production of ROS-scavenging enzymes, followed by the improved cell growth of keratinocytes. Based on our present results, well-designed animal and clinical studies will be needed for the potential translation of our preclinical findings in patients with oral cancer receiving chemotherapy and radiotherapy.

## Figures and Tables

**Figure 1:** Effects of 5-FU on the growth of (A) oral cancer (B88) cells and (B) oral keratinocytes (RT7). The cells were grown in 96-well plates in medium supplemented with 5-FU [0 (⋄), 1 (●), 2 (△), 5 (▲) and 10 (□) μg/ml] for 3 days. Viable cells were estimated by 3-(4,5-dimethylthi-azol-2-yl)-2,5-diphenyltetrazolium bromide (MTT) assay. The absorbance was measured at 570 nm. Standard deviations were calculated from three independent experiments. Growth was significantly lower compared to that in untreated cells. Although B88 cells were decreased in number by treatment with 5 and 10 μg/ml 5-FU, there was no apparent decrease in cell number when RT7 cells were treated with the same concentrations of 5-FU. Statistically significant at ^*^P<0.05 and ^**^P<0.01 (Mann-Whitney U test).

**Figure 2:** Effects of reactive oxygen species (ROS) on the growth of RT7 cells. (A) Generation of ROS in 5-FU-treated RT7 cells. The levels of ROS production were measured at 24 and 48 h after treatment of RT7 cells with 5-FU (10 μg/ml) using the ROS detection dye DCFH-DA. The total amount of ROS produced was significantly augmented at 48 h after treatment. (B) Effect of N-acetyl cysteine (NAC) on the generation of 5-FU-induced ROS. NAC (0.1 mM), a ROS scavenger, significantly suppressed the production of ROS at 48 h after treatment with 5-FU (10 μg/ml). (C) NAC improvement of cell growth in 5-FU-treated RT7 cells. Cells were treated with 5-FU (△), NAC (●), or both (▲). Combined treatment of RT7 cells with 5-FU (10 μg/ml) and NAC (0.1 mM) significantly recovered the impairment of cell growth as compared to the treatment with 5-FU alone. Statistically significant at ^*^P<0.05 (Mann-Whitney U test).

**Figure 3:** Effects of γ-tocotrienol on the growth and production of reactive oxygen species (ROS) in RT7 cells. (A) Cells were grown for 3 days in 96-well plates containing medium supplemented with 5-FU (10 μg/ml, △), γ-tocotrienol (γT3, 10 nM, ●), or both (▲). γ-tocotrienol treatment significantly restored the 5-FU-induced growth inhibition in RT7 cells. (B) Effect of γ-tocotrienol on the generation of 5-FU-induced ROS. γ-tocotrienol (γT3, 10 nM) significantly suppressed the production of ROS at 48 h after treatment with 5-FU (10 μg/ml). Statistically significant at ^*^P<0.05 and ^**^P<0.01 (Mann-Whitney U test).

**Figure 4:** Expression of the NF-E2-related factor 2 (Nrf2) protein and Kelch-like ECH-associated protein 1 (Keap1) in RT7 cells treated with 5-FU (10 μg/ml), γ-tocotrienol (γT3, 10 nM), or both. (A) Western blot analysis of Nrf2 protein present in the cytoplasm and nucleus in the cells treated with 5-FU, γ-tocotrienol, or both for 24 h. Cytosolic and nuclear extracts were subjected to western blot analysis to detect the expression levels of Nrf2 protein. Although 5-FU stimulated the nuclear localization of Nrf2 for up to 12 h after treatment, γ-tocotrienol had no effect on the cytoplasmic localization of Nrf2. On the other hand, simultaneous treatment of cells with both agents significantly stimulated the nuclear localization of Nrf2 for up to 24 h. As a loading control for the protein samples, the expression of β-actin is also shown. Results are representative of three independent experiments. (B) Western blot analysis for the detection of Keap1 in the cytoplasm. Cells were treated with 5-FU, γ-tocotrienol, or both for 24 h. Cytosolic fractions were analyzed for the detection of Keap1. Although 5-FU degraded the cytosolic Keap1 at 12 h after treatment, γ-tocotrienol had no effect on cytoplasmic localization of the Keap1. On the other hand, simultaneous treatment of cells with both agents significantly inhibited the cytoplasmic localization of Keap1 for up to 24 h. As a loading control for the protein samples, the expression of β-actin is also shown. Results are representative of three independent experiments. (C) Indirect immunofluorescence microscopy of Nrf2 protein in RT7 cells treated with or without (control, a–d) 5-FU (e–h), γ-tocotrienol (i–l), or both (m–p) for 24 h. The expression of activated Nrf2 was specifically observed in the nuclei of 5-FU-treated cells at 12 h (arrow, g). However, activated Nrf2 protein was continuously detected in the nuclei of the cells treated with both agents for 24 h (arrows, o and p).

**Figure 5:** Steady-state levels of (A) heme oxygenase-1 (HO-1) and (B) NAD(P)H:quinone oxidoreductase-1 (NQO-1) mRNA measured using quantitative real-time PCR. The primers and probes used for these experiments are described in the Materials and methods. The levels of HO-1 and NQO-1 mRNA expression in RT7 cells were compared with those (100%) under the basal condition. Each bar represents at least three separate mRNA isolations performed in duplicate. 5-FU treatment significantly enhanced the expression of HO-1 mRNA at 12 h, but HO-1 mRNA expression was remarkably inhibited by 5-FU at 24 h, indicating that the levels of HO-1 mRNA changed in parallel with the expression of NF-E2-related factor 2 (Nrf2) in 5-FU-treated cells. In contrast, combined treatment with 5-FU and γ-tocotrienol (γT3) resulted in the continuous enhancement of HO-1 mRNA expression in cells for up to 24 h. Similarly, NQO-1 mRNA expression was also regulated by 5-FU and γ-tocotrienol. Statistically significant at ^*^P<0.05 and ^**^P<0.01 (Mann-Whitney U test).
